The article "Pyrocatechol Alleviates Cisplatin-Induced Acute Kidney Injury by Inhibiting ROS Production" was published in 2022. Journal: Oxid Med Cell Longev.

# Pyrocatechol Alleviates Cisplatin-Induced Acute Kidney Injury by Inhibiting ROS Production

**DOI:** 10.1155/2022/2158644

**Published:** 2022-09-19

**Authors:** Xuexia Xie, Fan Wu, Jiaxin Tian, Zhilong Liu, Huibin He, Dongping Bao, Guoliang Li, Haomin Li, Jianfan Chen, Yiqi Lai, Zheng Chen, Jun Fan, Guo Chen, Caiyong Lai

**Affiliations:** ^1^Department of Urology, The First Affiliated Hospital of Jinan University, Guangzhou 510632, China; ^2^Department of Medical Biochemistry and Molecular Biology, Engineering Technology Research Center of Drug Development for Small Nucleic Acids, School of Medicine, Jinan University, Guangzhou 510632, China; ^3^Department of General Surgery, The First Affiliated Hospital, Jinan University, Guangzhou 510632, China; ^4^Department of Urology, Dongguan Kanghua Hospital, Dongguan, China; ^5^University of South China, Hengyang, China; ^6^School of Biopharmacy, China Pharmaceutical University, Nanjing 211198, China; ^7^Department of Urology, The Sixth Affiliated Hospital of Jinan University, Dongguan, China; ^8^Yang Xi General Hospital People's Hospital, Yangjiang, China

## Abstract

As one of the most common cancer chemotherapy drugs, cisplatin is widely used in cancer management. However, cisplatin-induced nephrotoxicity occurs in patients who receive this drug. This study is aimed at developing therapeutic agents that effectively alleviate the nephrotoxic effects during cisplatin treatment. We identified a compound named pyrocatechol (PCL) from a natural product library that significantly alleviated cisplatin-induced cytotoxicity *in vitro*. Pyrocatechol treatment substantially ameliorated cisplatin (20 mg · kg^−1^) treatment-induced neuropathological indexes, including inflammatory cell infiltration and apoptosis, *in vivo*. Mechanistically, pyrocatechol significantly prevented oxidative stress-induced apoptosis by activating glutathione peroxidase 4 (GPX4) to reduce reactive oxygen species (ROS) accumulation in cisplatin-treated cells. In addition, pyrocatechol significantly inhibited ROS-induced JNK/P38 activation. Thus, we found that pyrocatechol prevents ROS-mediated JNK/P38 MAPK activation, apoptosis, and cytotoxicity through GPX4. Our study demonstrated that pyrocatechol is a novel therapeutic agent against cisplatin-induced kidney injury.

## 1. Introduction

Cisplatin (dichloro diammine platinum) is one of the most commonly used and effective chemotherapy drugs, and it is widely used for the treatment of solid malignant tumors, such as head and neck, lung, ovarian, and bladder cancer [1, 2]. Despite its excellent antitumor activity, its application is hindered by a wide range of toxic side effects, such as nephrotoxicity, ototoxicity, neurotoxicity, and emetogenicity, of which nephrotoxicity is the most important sequela; renal dysfunction occurs in approximately one-third of cisplatin-treated patients [3, 4]. Therefore, how to alleviate cisplatin-induced kidney injury has become an urgent problem.

The article "Pyrocatechol Alleviates Cisplatin-Induced Acute Kidney Injury by Inhibiting ROS Production" was published in 2022. Journal: Oxid Med Cell Longev.

The main mechanisms by which cisplatin causes kidney injury include oxidative stress, necrosis, autophagy, and apoptosis [5]. Oxidative stress resulting from excessive production of reactive oxygen species (ROS) plays a critical role in cisplatin-induced kidney injury [6]. Cisplatin destroys intracellular antioxidants, disrupts the redox balance, and interferes with the mitochondrial respiratory chain, leading to elevated ROS [7]. Many studies have reported that excess ROS induce the JNK/P38 MAPK signaling pathway and activate caspase-dependent apoptosis [8, 9]. Glutathione peroxidase 4 (GPX4) is a ubiquitously expressed, glutathione- (GSH-) dependent enzyme that plays a central role in counteracting ROS-mediated cytotoxicity. Moreover, inactivation of GPX4 was reported to lead to intracellular ROS accumulation [10].

This study was aimed at exploring small molecule drugs that could alleviate the nephrotoxic effects of cisplatin. We screened a natural product library of 1600 compounds and identified a compound called pyrocatechol that significantly attenuated cisplatin-induced cytotoxicity. Pyrocatechol is a small naturally occurring compound in plants such as *Bonellia macrocarpa*, *Semecarpus anacardium*, onions, apples, and olive oil [11, 12]. This compound has been utilized in the management of various cancers, including glioblastoma [13], lung cancer cells [14], and breast cancer cells [15]. Pyrocatechol has also been reported to exert anti-inflammatory, antiapoptotic, and antioxidant activities [16–18].

However, the effects of pyrocatechol on cisplatin-induced nephrotoxicity and its molecular mechanism remain unknown. In this study, we investigated the beneficial effects of pyrocatechol on cisplatin-induced kidney injury *in vivo* and *in vitro*. At the molecular level, pyrocatechol directly inhibited apoptosis by regulating the ROS-JNK/P38 MAPK signaling pathway in a GPX4-dependent manner. In conclusion, this study demonstrates for the first time that pyrocatechol has a significant protective effect against cisplatin-induced renal injury by impeding apoptosis, revealing its target of action.

## 2. Materials and Methods

### 2.1. Animal Experiments

Male C57BL/6 mice (8-10 weeks, 20-25 g) were purchased from Yancheng Biotechnology Company (Guangzhou, China). All experimental procedures were approved by the Institutional Animal Care and Use Committee of Jinan University. Mice were fed under standard conditions. After one week of adaptation to feeding conditions, the mice were injected intraperitoneally with cisplatin (20 mg · kg^−1^) to induce a model of kidney injury. The mice were divided into four groups: control, cisplatin (20 mg · kg^−1^), cisplatin (20 mg · kg^−1^) + pyrocatechol (30 mg · kg^−1^), and pyrocatechol (30 mg · kg^−1^) [14, 19, 20]. Pyrocatechol was injected intraperitoneally 6 hours before cisplatin injection and administered daily. The control group was given saline only. After three days, all animals underwent cervical dislocation, and blood and kidney samples were collected for further experiments.

The article "Pyrocatechol Alleviates Cisplatin-Induced Acute Kidney Injury by Inhibiting ROS Production" was published in 2022. Journal: Oxid Med Cell Longev.

### 2.2. Cell Culture and Treatment

HEK293T cells were purchased from the American Type Culture Collection (ATCC) and cultured in DMEM (Gibco) with 10% FBS (Excell, Shanghai, China), 100 U/mL penicillin (Vivacell, Shanghai, China), and 100 U/mL streptomycin. HK-2 cells were obtained from the China Cell Bank and were maintained in DMEM/Ham's F12 (BI) with 5% fetal bovine serum (BI). All the cells were cultured in 37°C incubators with 5% CO_2_. Cells were treated with various concentrations of cisplatin, pyrocatechol, and other drugs for 24 hours.

### 2.3. Hematoxylin and Eosin (H&E) Staining

Kidney tissues from mice were embedded in paraffin and cut into sections. Then, the sections were stained with hematoxylin and eosin (H&E). A semiquantitative score was used for renal tubular injury; 0 corresponded to 0% injury or 0.5% to <10% injury, 1 to 10-25% injury, 2 to 2-50% injury, 3 to 51-75% injury, and 4 to 76-100% injury. At least six renal regions were randomly selected for each slide under the microscope.

### 2.4. Terminal Transferase dUTP Nick-End Labeling (TUNEL) Assay

The TUNEL assay was used to assess cell death in mouse kidney tissue. Briefly, kidney tissue sections were dewaxed in xylene and ethanol, washed in PBS, and then incubated with a concentration of 20 *μ*g/mL of Nase K-free protease for 15 minutes at room temperature, followed by three washes in PBS or HBSS. The sections were then incubated with the TUNEL reaction mixture for 2 hours at 4°C. The kidney tissue of the mice was observed with a microscope and photographed.

### 2.5. Renal Functional Parameters

Blood creatinine and blood urea nitrogen levels in mice were measured using a colorimetric kit (C011-2-1, Nanjing Jiancheng Institute of Biological Engineering, Nanjing, China) and an enzymatic assay kit (C013-2-1, Nanjing Jiancheng Institute of Biological Engineering, Nanjing, China), respectively, according to the protocol provided by the manufacturer. Mouse renal function was assessed based on measured blood creatinine and urea nitrogen levels in mice.

The article "Pyrocatechol Alleviates Cisplatin-Induced Acute Kidney Injury by Inhibiting ROS Production" was published in 2022. Journal: Oxid Med Cell Longev.

### 2.6. Cell Counting Kit-8 (CCK-8) Assay

Cell viability was determined using the CCK-8 assay. Cells were cultured in 96-well plates and treated with the drug. After treatment, the CCK-8 reagent (10 *μ*L; Dojindo) was added to the cell culture medium. After incubation in an incubator at 37°C for 1 hour, the absorbance of cells from different study groups was measured at 450 nm using an enzyme marker.

### 2.7. GSH Assay

GSH concentrations in mouse kidney lysates were measured using a GSH assay kit purchased from Nanjing Jiancheng Bioengineering Institute (Nanjing, China) following the instructions for the reagents.

### 2.8. MDA Assay

Malondialdehyde (MDA) is one of the end products of lipid peroxidation, and concentrations were assessed in mouse kidney lysates using a lipid oxidation (MDA) assay kit purchased from Beyotime Biotechnology (Shanghai, China) according to the manufacturer's instructions. The manufacturer's instructions were followed to measure renal lipid peroxidation.

### 2.9. Intracellular ROS Measurement

Intracellular ROS levels were measured by the DCF method. After treatment, cells were collected using a PPS wash, followed by an examination of intracellular ROS levels using 2′,7′-dichlorofluorescein diacetate (H2DCF-DA, Thermo Fisher Scientific). Cells were incubated with DCFH-DA (20 *μ*M) for 30 minutes at room temperature in the dark, washed three times with PBS, and evaluated using an Eisen Biologics flow cytometer (Novocyte 2060r) to measure intracellular ROS levels.

### 2.10. SOD and CAT Assay

Cells were harvested with 0.25% trypsin and washed twice with PBS. Then, the cellular activities of superoxide dismutase (SOD) and catalase (CAT) were determined using the CAT Assay Kit (Beyotime, Shanghai, China) and Total Superoxide Dismutase Assay Kit with WST-8 (Beyotime, Shanghai, China) according to the manufacturer's instructions. Briefly, the SOD assay was performed by mixing 20 *μ*L of protein sample with 160 *μ*L of WST-8 enzyme working solution and 20 *μ*L of diluted reaction start working solution and then incubated at 37°C for 30 minutes. After reaction, the absorbance of the sample was measured at 450 nm, while the CAT assay kit is performed by mixing 36.5 *μ*L of Catalase Assay Buffer with 3.5 *μ*L of protein sample and then incubated with 10 *μ*L of 250 mM hydrogen peroxide solution. 10 *μ*L of the above samples was mixed with 200 *μ*L of coloring working solution and incubated for 15 minutes. After reaction, the absorbance of the sample was measured at 520 nm.

### 2.11. Real-Time PCR Analysis

Total RNA was extracted from tissues or cells using the Total RNA Extraction Kit (R1200, Solarbio) following the manufacturer's instructions. cDNA was extracted using a reverse transcription kit (Vazyme, Nanjing, China). qRT-PCR was performed with the SYBR Green Real-Time PCR Master Mix (Vazyme, Nanjing, China). Actin was used as a standard control. The relative RNA expression levels were calculated using the 2^−*ΔΔ*CT^ method. All primers were custom-made by Sangon Biotech.

The article "Pyrocatechol Alleviates Cisplatin-Induced Acute Kidney Injury by Inhibiting ROS Production" was published in 2022. Journal: Oxid Med Cell Longev.

### 2.12. Annexin V/PI Double Staining

After HK-2 cells were treated for 24 hours, the cells were digested with trypsin, washed with PBS, and transferred to flow cytometry tubes. Cells were coincubated with Annexin V-Fluorescein Isothiocyanate (FITC) and PI for 5 minutes in the dark. Apoptotic cells were detected by flow cytometry.

### 2.13. Western Blotting

A lysis buffer (RIPA, Beyotime, China) was added to each group of cells or tissues to fully lyse and extract total protein from the cells. Lysates were electrophoresed on 6-12% gels using sodium dodecyl sulfate (SDS) polyacrylamide gel electrophoresis (PAGE). Protein isolates were transferred to PVDF membranes (Millipore, USA) and blocked in 5% skim milk powder solution for 1 h at room temperature. The cells were incubated with primary antibody overnight at 4°C. Primary antibodies against GPX4 (Proteintech, USA), B-cell lymphoma-2 (Bcl-2) (Abcam, USA), Cleaved Caspase-3 (CST, USA), p-ERK (CST, USA), ERK (CST, USA), p-p38 (CST, USA), p38 (CST, USA), p-JNK (CST, USA), JNK (CST, USA), and *β*-actin (Santa Cruz, USA) were used. The appropriate secondary antibody (1 : 5000; Cell Signaling Technology, USA) was incubated for 1 hour at 37°C on a shaker, and the bands were observed using ECL chemiluminescence (Beyotime Biotechnology, China). ImageLab software was used for data analysis.

### 2.14. RNA Interference

HK-2 cells were cultured and then infected with GPX4-shRNA lentivirus for 72 hr. HK-2 cells were screened with puromycin (Beyotime Biotechnology, China). Single-cell clones resistant to puromycin were amplified and screened by western blotting using an anti-GPX4 antibody (1 : 1,000, Beyotime Biotechnology, China).

### 2.15. Statistical Analysis

SPSS 26.0 and GraphPad Prism 7 software were used for statistical analysis. All measurements were tested for normality and homogeneity of variance, and the data are presented as the mean ± SEM. Differences between two or more groups were assessed by performing Student's *t* test and one-way ANOVA. *P* < 0.05 indicates that the differences are statistically significant.

## 3. Results

### 3.1. Pyrocatechol Alleviates Cisplatin-Induced AKI

To identify compounds that alleviate cisplatin-induced cytotoxicity, we performed chemical screening using a natural product library consisting of approximately 1600 representative compounds. Renal epithelial cells (HK-2) were treated with cisplatin in the presence or absence of each compound in the library for 48 hours, and cell viability was determined using the CCK-8 assay (Figure 1(a)). With this screening strategy, pyrocatechol was found to significantly inhibit cisplatin-induced cytotoxicity (Figure 1(b)). Cotreatment with pyrocatechol and cisplatin significantly increased the viability of renal cells, including HK-2 and H293T cells, compared with cisplatin treatment alone (Figures 1(c) and 1(d)).

The article "Pyrocatechol Alleviates Cisplatin-Induced Acute Kidney Injury by Inhibiting ROS Production" was published in 2022. Journal: Oxid Med Cell Longev.

### 3.2. Pyrocatechol Exerts a Protective Effect on Apoptosis *In Vitro*

Cisplatin causes apoptotic cell death in various types of cells, which is attributed to its cytotoxicity [21, 22]. Hence, we examined whether pyrocatechol could prevent cisplatin-induced apoptosis in HK-2 and 293T cells. As shown in Figure 2(a), we found that pyrocatechol treatment completely abolished cisplatin-induced cell death. Moreover, annexin V staining analysis showed that cisplatin induced apoptosis in 25 ± 2.4% of HK-2 cells, while the combination of pyrocatechol and cisplatin reduced the number of apoptotic cells to 9 ± 2.8% (Figure 2(b)). In addition, western blot analysis showed that cisplatin treatment significantly reduced the Bcl-2 protein expression and increased the level of the Cleaved Caspase-3 protein. However, pyrocatechol almost completely blocked the reduction in Bcl-2 and Caspase-3 cleavage in HK-2 cells (Figure 2(c)).

### 3.3. Effect of Pyrocatechol on Oxidative Stress in Cisplatin-Treated HK-2 Cells

Oxidative stress was reported to be the main mechanism for cisplatin-induced apoptosis [23]. To investigate the level of intracellular ROS, we next used the sensitive fluorescent probe DCFH-DA to label the ROS in cells. The results showed a significant increase in intracellular ROS levels in the cisplatin-treated cells. However, pyrocatechol reversed the increase in ROS (Figure 3(a)). We then investigated the level of glutathione, which is a major antioxidant in the mitigation of cisplatin nephrotoxicity [24, 25]. The results showed that compared with the control, cisplatin could significantly reduce the glutathione level in HK-2 cells. However, pyrocatechol reversed the cisplatin-induced decrease in GSH levels (Figure 3(b)). We next examined the protein expression of GPX4, which is a GSH-dependent enzyme that inhibits the production of ROS. As shown in Figure 3(c), cisplatin treatment significantly reduced the expression of GPX4 protein. However, pyrocatechol almost completely restored the protein expression level of GPX4. These findings support the hypothesis that pyrocatechol can substantially alleviate oxidative stress induced by cisplatin-induced renal injury.

The article "Pyrocatechol Alleviates Cisplatin-Induced Acute Kidney Injury by Inhibiting ROS Production" was published in 2022. Journal: Oxid Med Cell Longev.

### 3.4. Pyrocatechol Alleviates Cisplatin-Induced Apoptosis through P38/JNK Pathway

To further verify the protective mechanism of pyrocatechol in cisplatin-induced apoptosis, we analyzed the MAPK-related signaling pathway by western blotting. The results are shown in Figure 4(a). Pyrocatechol attenuated the levels of p-JNK and p-p38 in the cisplatin-treated HK-2 cells. However, pyrocatechol did not affect the level of p-ERK. Moreover, we found that NAC (N-acetyl-l-cysteine), an ROS scavenger, could block cisplatin-induced JNK and p38 activation (Figure 4(b)). These results suggest that cisplatin activates the MAPK signaling pathway through stimulation of ROS production, thereby inducing apoptosis.

We further used anisomycin (a specific activator of P38/JNK) to explore the roles of P38/JNK activation in pyrocatechol-mediated inhibition of cisplatin-induced HK-2 cell apoptosis. Interestingly, the results showed that anisomycin reversed the inhibitory effect of pyrocatechol on the expression of p-JNK and p-p38, as well as Cleaved Caspase-3, in the cisplatin-treated cells (Figure 4(c)). Moreover, analysis of apoptosis by annexin V staining showed that anisomycin reversed the antiapoptotic effect of pyrocatechol on cisplatin-treated cells (Figure 4(d)). These results suggest that pyrocatechol alleviates cisplatin-induced apoptosis through the P38/JNK pathway.

### 3.5. Pyrocatechol Reduces ROS Accumulation Induced by Cisplatin in HK-2 Cells in a GPX4-Dependent Manner

We found that pyrocatechol could block the cisplatin-induced GPX4 reduction (Figure 3(c)). We hence speculate that pyrocatechol exerts its protective effects on ROS-mediated cytotoxicity, including cell apoptosis and MAPK activation, through GPX4. To test this hypothesis, we used the CRISPR/Cas9 technique to knock out the expression of endogenous GPX4 in HK-2 cells (Figure 5(a)). As expected, we found that pyrocatechol could not restore cisplatin-mediated inhibition of GPX4 knockout (GPX4-KO) cell viability (Figure 5(b)). Furthermore, pyrocatechol could not inhibit cisplatin-induced elevation of ROS production in the GPX4 knockout cells (Figure 5(c)). The above results suggest that the GPX4 protein plays a vital role in the effect of pyrocatechol on cisplatin-induced AKI.

### 3.6. Pyrocatechol Protects against Cisplatin-Induced AKI in Mice

A mouse model of cisplatin-induced kidney injury was used to investigate whether pyrocatechol could alleviate cisplatin-induced nephrotoxicity. Cisplatin (20 mg·kg^−1^) was injected intraperitoneally to induce kidney damage in mice according to the experimental design (Figure 6(a)). The treatment group received oral administration of pyrocatechol (30 mg·kg^−1^) 6 hours before cisplatin injection and continued daily administration once after cisplatin treatment. Pathological analysis of the mouse kidney injury score showed that pyrocatechol significantly alleviated cisplatin-induced AKI in mice (Figure 6(c)). Moreover, treatment with pyrocatechol reversed the cisplatin-induced increase in SCr and BUN levels (Figure 6(b)). To examine the protective effect of pyrocatechol on cisplatin-induced histopathological damage to the kidney, we stained mouse kidney sections with H&E. As shown in Figure 6(d), the kidneys of the cisplatin-treated mice showed severe damage with inflammatory cell infiltration and tissue vacuolation. However, renal tissue tubular damage was significantly relieved in the pyrocatechol and cisplatin combination-treated mice. More importantly, the serum creatinine and blood urea nitrogen from the mice that received pyrocatechol alone showed no significant change compared with those from the control mice. Furthermore, H&E staining of the kidneys showed that pyrocatechol did not induce nephrotoxicity.

The article "Pyrocatechol Alleviates Cisplatin-Induced Acute Kidney Injury by Inhibiting ROS Production" was published in 2022. Journal: Oxid Med Cell Longev.

To further explore the roles of pyrocatechol in cisplatin-induced nephrotoxicity, we investigated the mRNA expression of kidney injury molecule-1 (KIM-1) and neutrophil gelatinase-associated lipocalin (NGAL), two known tubular biomarkers of early kidney injury [26]. The results showed (Figure 6(e)) that the expression levels of KIM-1 and NGAL were significantly increased in the cisplatin-injured kidneys. However, combined treatment with cisplatin and pyrocatechol significantly reversed the increase in KIM-1 and NGAL expression. Klotho is mainly expressed in the distal convoluted tubules of the kidney and has anti-inflammatory and antioxidant properties. The onset of acute kidney injury is usually accompanied by low levels of klotho [27]. We further evaluated klotho expression, and the results showed that klotho expression was decreased in the cisplatin-treated group. However, cotreatment with cisplatin and pyrocatechol significantly alleviated the loss of klotho caused by cisplatin-induced acute kidney injury. In conclusion, pyrocatechol was effective in protecting against cisplatin-induced renal injury.

### 3.7. Effects of Pyrocatechol on the Cisplatin-Induced Inflammatory Response and Oxidative Stress

The inflammatory response is one of the major causes of cisplatin-induced acute kidney injury [28]. To investigate the effect of pyrocatechol on the inflammatory response in mouse renal tubular cells, we examined the expression of proinflammatory cytokines, including IL-6 and TNF-*α*, in each group. The results showed (Figures 7(a) and 7(b)) that the mRNA levels of the inflammatory factors IL-6 and TNF-*α* were significantly increased in the cisplatin-treated group; however, cotreatment with pyrocatechol significantly attenuated the increase in cisplatin-induced inflammatory factors. In addition, the increased expression of chemokines, including C–C motif chemokine ligand 2 (CCL2/MCP-1), TNF superfamily member 12A (TWEAK receptor; TNFRSF12A; Fn14), and TNF superfamily member 12 (TWEAK; TNFSF12), during cisplatin treatment was significantly suppressed by pyrocatechol (Figures 7(c)–7(e)). Therefore, the above results demonstrated that pyrocatechol significantly attenuated the cisplatin-induced inflammatory response.

The article "Pyrocatechol Alleviates Cisplatin-Induced Acute Kidney Injury by Inhibiting ROS Production" was published in 2022. Journal: Oxid Med Cell Longev.

Previous reports showed that cisplatin could significantly reduce glutathione, superoxide dismutase, and catalase activities in renal tissue [29]. We hence examined the levels of superoxide dismutase and catalase; compared with the cisplatin group, we found that the pyrocatechol treatment group significantly increased glutathione levels, but did not reverse cisplatin-induced reductions in superoxide dismutase and catalase activities (Figures 7(f)–7(h)). We further examined the protein expression of GPX4. As shown in Figure 7(i), cisplatin treatment significantly reduced the expression of GPX4 protein. Intriguingly, pyrocatechol almost restored the protein expression level of GPX4. Previous studies reported that GSH is the primary detoxification mechanism of cisplatin nephrotoxicity [30, 31]. Therefore, the results in Figure 7 show that pyrocatechol alleviates oxidative stress induced by cisplatin-induced renal injury mainly by reversing GSH and GPX4 levels.

### 3.8. Pyrocatechol Ameliorates Acute Renal Injury in Cisplatin-Treated Mice by Inhibiting Apoptosis

Kidney cells often undergo apoptotic cell death during renal injury [32]. We next analyzed apoptosis by examining Bcl-2 and Cleaved Caspase-3, which are hallmarks of apoptosis, to further clarify the role of apoptosis in cisplatin-induced kidney injury *in vivo*. As shown in Figure 8(a), cisplatin treatment significantly reduced the expression of Bcl-2 protein and increased the expression of Cleaved Caspase-3, indicating that cisplatin induces kidney cell apoptosis. However, cotreatment with pyrocatechol fully restored the changes in these proteins. Moreover, the TUNEL assay further revealed that pyrocatechol could significantly diminish the cisplatin-induced increase in the number of TUNEL-positive cells in kidney tissues (Figure 8(b)), indicating that pyrocatechol exerted a beneficial effect on cisplatin-induced kidney injury by inhibiting apoptosis in mice. In summary, pyrocatechol exerted a beneficial effect on cisplatin-induced kidney injury by inhibiting apoptosis (Figure 8(c)).

The article "Pyrocatechol Alleviates Cisplatin-Induced Acute Kidney Injury by Inhibiting ROS Production" was published in 2022. Journal: Oxid Med Cell Longev.

## 4. Discussion

Cisplatin is one of the most widely used chemotherapeutic drugs, and AKI is the main side effect of cisplatin-based therapy [33]. Approximately one-third of patients treated with cisplatin develop renal dysfunction. According to earlier reports, the main mechanisms of cisplatin-induced acute kidney injury (AKI) include oxidative stress, inflammation, and apoptosis [5]. We aimed to explore compounds that alleviate the nephrotoxic effects of cisplatin. First, we found a natural product called pyrocatechol, which could alleviate cisplatin-induced nephrotoxicity, by screening a library of 1600 natural products. Pyrocatechol is a small naturally occurring compound present in plants, including *B. macrocarpa*, *S. anacardium*, onions, apples, and olive oil [12]. Earlier studies have shown that pyrocatechol has a potent antioxidant and anti-inflammatory effect in various human diseases [18, 20]. In our current study, we aimed to investigate the protective effect of pyrocatechol on cisplatin-induced nephrotoxicity *in vitro* and *in vivo*.

Our study demonstrated that pyrocatechol significantly alleviates cisplatin-induced nephrotoxicity in mice. This protective effect of pyrocatechol on kidney injury was manifested by a reduction in renal tubular apoptosis, an improvement in the renal tubular inflammatory response, and an increase in the antioxidant capacity of the kidney. In our study, we tested pyrocatechol *in vivo* at a dose of 20 mg · kg^−1^. The *in vivo* experiments showed that treatment with pyrocatechol alone did not cause significant adverse effects in mice. At this safe dose, pyrocatechol significantly reduced serum creatinine and blood urea nitrogen levels in the cisplatin-treated mice and reversed inflammation in the mice. Therefore, pyrocatechol is a safe and effective drug candidate for cisplatin-induced AKI.

Cisplatin accumulates as a highly active metabolite in renal epithelial cells, disrupting renal cell antioxidant functions, which consequently leads to ROS accumulation and causes mitochondrial impairment [34, 35]. In this study, we demonstrate that pyrocatechol significantly inhibits the elevation of ROS levels and oxidative stress induced by cisplatin-induced renal injury *in vivo* and *in vitro* by reversing the changes in GSH and GPX4. Renal tissue damage, characterized by tubular cell death, is a common histopathological feature of cisplatin nephrotoxicity [3]. Under this condition, apoptosis is the primary type of tubular programmed cell death. Our results showed that apoptosis in cisplatin-treated mouse kidney tissue was significantly attenuated.

The article "Pyrocatechol Alleviates Cisplatin-Induced Acute Kidney Injury by Inhibiting ROS Production" was published in 2022. Journal: Oxid Med Cell Longev.

Dysregulation of ROS levels leading to oxidative stress plays a crucial role in cisplatin-induced kidney injury. Cisplatin is reported to increase free radical levels to induce cell death [36]. ROS activate antioxidant systems including GSH and SOD, which subsequently reduces ROS-induced oxidative damage [37]. Meanwhile, the activation of the antioxidant system such as GSH, SOD, and glutathione peroxidase is also recognized as the biomarkers for oxidative stress [38]. In another way, the severe impairment of antioxidant enzymes such as GSH, SOD, catalase, and GPXs is also important indicators to ascertain the oxidative stress index [39, 40]. For instance, MDA is rapidly overproduced in response to lipid peroxidation and is usually accompanied with GPX4 reduction [41]. In the present study, our data showed that cisplatin treatment significantly decreased GSH, catalase, and SOD activity, indicating that server oxidative stress is induced by cisplatin treatment. However, pyrocatechol could reverse the reduction of these antioxidant enzymes caused by cisplatin treatment. These data provide evidences that pyrocatechol potently alleviated cisplatin-induced oxidative stress. In addition, cisplatin-induced increases in ROS levels damage mitochondria and activate mitogen-activated protein kinases (MAPKs), including p38, c-Jun N-terminal kinase (JNK), and extracellular signal-regulated kinase 1/2 (ERK1/2), thereby inducing apoptosis [42–44]. In our study, pyrocatechol alleviates cisplatin-induced apoptosis through the P38/JNK pathway. Anisomycin, a specific activator of p38/JNK [45], reverses the inhibitory effect of pyrocatechol on the expression of p-JNK, p-p38, and the apoptotic protein Cleavage Caspase-3 in cisplatin-induced cells.

GPX4 is a selenocysteine-containing peroxidase enzyme catalyzing reduction of toxic peroxides, organic hydroperoxides, and lipid hydroperoxides into respective nontoxic alcohols [46]. GPX4 belongs to the glutathione peroxidase family member protein, which is a central component of the cellular antioxidation system and uses reduced glutathione (GSH) as a reducing agent [47, 48]. As one of the main antioxidant mediators, GPX4 plays an important role in regulation of oxidation-induced cell death, and it is considered as the main suppressor of ferroptosis, a cell death induced by lipid peroxidation [10]. Our study demonstrated that pyrocatechol almost completely restored cisplatin-induced reduction of cellular GPX4 protein expression. And we proved that pyrocatechol could alleviate cisplatin-induced apoptosis by affecting the expression level of GPX4 and regulating the ROS/P38/JNK pathway. Our study indicated that the pyrocatechol-induced decrease in intracellular ROS generation in cisplatin-treated cells was completely inhibited by GPX4 knockdown. Therefore, the possible mechanism by which pyrocatechol induces cisplatin-induced kidney injury is that pyrocatechol activates GPX4 and regulates the ROS/JNK/p38 MAPK signaling pathway to protect the kidney.

The article "Pyrocatechol Alleviates Cisplatin-Induced Acute Kidney Injury by Inhibiting ROS Production" was published in 2022. Journal: Oxid Med Cell Longev.

## 5. Conclusion

In conclusion, our findings suggest that pyrocatechol has a protective effect against cisplatin-induced renal injury by attenuating oxidative stress, inflammation, and apoptotic pathways. This protective effect was mainly through activation of GPX4, inhibition of the ROS/JNK/p38 MAPK signaling pathway, and then modulation of apoptosis to protect the kidney. This result provides a basis for the clinical treatment of cisplatin-induced AKI, and further validation of the molecular mechanism of apoptosis inhibition by pyrocatechol is necessary.

## Figures and Tables

**Figure 1:** Pyrocatechol inhibits the cytotoxicity of cisplatin. (a) Screening for compounds that inhibit cytotoxicity in the presence of cisplatin was determined using the CCK-8 assay. (b) Chemical structure of the target compound pyrocatechol. (c, d) Pyrocatechol is protective against cisplatin-induced cytotoxicity. HK-2 and 293T cells were treated with cisplatin (20 *μ*M) to observe the changes in cell viability after 24 h of pyrocatechol action at different concentrations. Data are presented as means ± the standard deviation (*n* = 3). Data were normalized to the vehicle condition.

**Figure 2:** Pyrocatechol exerts a protective effect on apoptosis in vitro. (a) Representative microscopic images showing cytotoxicity after 24 hours of treatment of HK-2 and 293T cells with drugs. (b) Flow cytometry analysis of apoptosis results of pyrocatechol on cisplatin-treated HK-2 cells. (c) The expression levels of apoptosis-associated proteins B-cell lymphoma 2 (Bcl-2) and Cleaved Caspase-3 in HK-2 cells by western blotting. Values are presented as the means ± SD (*n* = 3). The statistical analysis was performed with two-way ANOVA.

**Figure 3:** (a) Cellular ROS levels were examined with H2DCF-DA using flow cytometry. (b) The effect of pyrocatechol on glutathione (GSH) levels was evaluated in HK-2 cells. (c) The expression of glutathione peroxidase 4 (GPX4) in HK-2 cells was measured. Values are presented as the means ± SD (*n* = 3). The statistical analysis was performed with two-way ANOVA.

**Figure 4:** Pyrocatechol alleviates cisplatin-induced apoptosis through P38/JNK pathway. (a) Western blotting was used to measure the expression of MAPK pathway proteins after treatment with cisplatin and pyrocatechol. The expression of MAPK pathway proteins, including p38, p-p38, c-Jun N-terminal kinase (JNK), p-c-Jun N-terminal kinase (p-JNK), extracellular signal-regulated kinase (ERK), and p extracellular signal-regulated kinase (p-ERK). (b) Western blotting was used to measure the expression of MAPK pathway proteins after treatment with cisplatin and ROS inhibitor (NAC, N-Acetyl-L-cysteine). (c) Western blotting was used to measure the expression of proteins treated with the P38/JNK agonist anisomycin, including p38, p-p38, JNK, p-JNK, and Cleaved Caspase-3. (d) Flow cytometric analysis of apoptosis in anisomycin-treated HK-2 cells. Values are presented as the means ± SD (*n* = 3). The statistical analysis was performed with two-way ANOVA.

The article "Pyrocatechol Alleviates Cisplatin-Induced Acute Kidney Injury by Inhibiting ROS Production" was published in 2022. Journal: Oxid Med Cell Longev.

**Figure 5:** The antiapoptotic effect of pyrocatechol is dependent on glutathione peroxidase 4 (GPX4). (a) The knockout efficacy was investigated using western blotting. (b) GPX4-KO HK-2 cells were treated with cisplatin (20 *μ*M) in the absence or presence of pyrocatechol for 24 hours, and cell viability was then determined. (c) GPX4-KO HK-2 cells were treated with cisplatin (20 *μ*M) in the absence or presence of pyrocatechol for 24 hours, and then, their ROS levels were measured by flow cytometry. Values are presented as the means ± SD (*n* = 3). The statistical analysis was performed with two-way ANOVA.

**Figure 6:** Pyrocatechol protects against cisplatin-induced nephrotoxicity in vivo. (a) Schematic design of animal experiments showing mice induced with cisplatin or pretreated with pyrocatechol. (b) Blood urea nitrogen (BUN) and serum creatinine levels between the treatment groups. The four groups of mice were treated differently according to the experimental design chart. (c, d) The low panel shows semiquantitative scores for tubular injury (c); a micrograph of a representative H&E-stained kidney section after hematoxylin and eosin (H&E) staining (d). Scale bars, 50 *μ*M. (e) The levels of the renal injury molecule-1 (KIM-1), neutrophil gelatinase-associated lipocalin (NGAL), and klotho mRNAs in kidney tissue were measured using real-time PCR. Data are presented as means ± the standard deviation (*n* = 6). The statistical analysis was performed with one-way ANOVA.

**Figure 7:** Effects of pyrocatechol on cisplatin-induced inflammatory response and oxidative stress. (a, b) The levels of TNF-*α* and IL-6 in kidney tissue were measured using real-time PCR. (c–e) The levels of multiple chemokines, such as C–C motif chemokine ligand 2 (MCP-1), TNF superfamily member 12A (Fn14), and TNF superfamily member 12 (TWEAK), in kidney tissue was measured using real-time PCR. (f) The effect of pyrocatechol on glutathione (GSH) levels was evaluated. (g) The effect of pyrocatechol on superoxide dismutase (SOD) levels was evaluated. (h) The effect of pyrocatechol on catalase levels was evaluated. (i) Expression of glutathione peroxidase 4 (GPX4) in pyrocatechol-treated kidney tissue lysates by western blotting. Data are presented as means ± the standard deviation (*n* = 6). The statistical analysis was performed with one-way ANOVA.

The article "Pyrocatechol Alleviates Cisplatin-Induced Acute Kidney Injury by Inhibiting ROS Production" was published in 2022. Journal: Oxid Med Cell Longev.

**Figure 8:** Pyrocatechol mitigated apoptosis in cisplatin-injured kidneys. (a) Expression of apoptosis-associated proteins B-cell lymphoma 2 (Bcl-2) and Cleaved Caspase-3 in pyrocatechol-treated kidney tissue lysates by Western blotting. (b) Representative images of TUNEL staining tests in kidney tissue. Scale bar, 100 *μ*M. Quantification of the number of positive cells assessed for TUNEL staining. Data are presented as means ± the standard deviation (*n* = 6). (c) Schematic diagram illustrating PCL inhibition of cisplatin-mediated apoptosis upregulating GPX4 to regulate AKI. The statistical analysis was performed with one-way ANOVA.

## Data Availability

The data that support the findings of this study are available from the corresponding authors upon reasonable request. Some data may not be made available because of privacy or ethical restrictions.
